The article "Long Noncoding RNA NORAD Promotes Fracture Healing through Interacting with Osteoblast Differentiation via Targeting miR-26a" was published in 2023. Journal: Biomed Res Int.

# Long Noncoding RNA NORAD Promotes Fracture Healing through Interacting with Osteoblast Differentiation via Targeting miR-26a

**DOI:** 10.1155/2023/9950037

**Published:** 2023-01-23

**Authors:** Siyuan Chen, Huili Ma, Mintao Li, Zhuting Jia, Xi Chen, Naitong Bu

**Affiliations:** ^1^Surgery of Spinal Degeneration and Deformity, Affiliated Hospital of Guangdong Medical University, Zhanjiang 524000, China; ^2^Department of Emergency Surgical Trauma Center, BinZhou Medical University Hospital, Binzhou 256603, China

## Abstract

The present study was designed to evaluate the dynamic expression of lncRNA NORAD in fracture healing of patients with brittle fractures and explore the function and mechanism of NORAD in regulating osteoblastic proliferation, differentiation, and apoptosis. The expression level of NORAD was detected by quantitative real-time PCR. The proliferation, differentiation, and apoptosis of osteoblasts were analyzed by MTT assay, ELISA, and flow cytometry. Luciferase report analysis was used to confirm the interaction between NORAD and its target ceRNA miR-26a. This study showed no significant differences in serum NORAD expression on the 7th day during fracture healing in patients, but increased expression of NORAD was certified on the 14, 21, and 28 days after fixation. Overexpression of NORAD promoted the proliferation and differentiation of osteoblasts and suppressed the apoptosis of osteoblasts. miR-26a proved to be the target gene of NORAD and was inhibited by overexpression of NORAD in osteoblasts. The enhanced expression of miR-26a was negatively linked to the lessened expression of NORAD. NORAD could accelerate the proliferation and differentiation of osteoblasts and inhibit apoptosis, thereby promoting fracture healing.

## 1. Introduction

Osteoporosis (OP) is one kind of endocrine disorder characterized by decreased bone mineral density, damaged bone microstructures, and osteopenia, which often occurs in the elderly [1]. Brittle fracture is a common clinical symptom of osteoporosis [2, 3]. In spite of the fact that fractures have a certain recuperating capacity, there are still 5%-10% of patients with fractures who have deferred or nonhealing problems, which leads to limited strolling and incessant torment, severe impair patients' life quality, and brings a tremendous burden to patients [4]. Fracture healing is a complex and moderate process of regeneration regulated by a variety of cytokines and stimulants [5]. Fracture healing could be a complex and moderate status of recovery controlled by an assortment of cytokines and stimulants. Osteoblast and osteoclast formation, apoptosis rate, and maintenance play a key role in fracture healing [6]. If there are problems with the proliferation, differentiation, and apoptosis of osteoblasts, the balance between bone formation and bone resorption will destroy, thus, bone healing will fail [7]. Therefore, it is important to study the exact mechanism of fracture occurrence and bone regeneration.

lncRNAs are endogenous noncoding RNA molecules that affect numerous biological activities. lncRNAs are involved in the management of mRNAs' expression, influencing different organic processes, like bone metabolism [8]. lncRNA KCNQ1OT1 is lowly expressed in individuals with intractable fracture healing, indicating its function in predicting delayed fracture [9]. GAS5 serves as a beneficial target in osteoporosis, which is exhibited by facilitating osteoblast differentiation [10]. NORAD is a widely researched lncRNA because of its function on diseases, cell cycles, and therapeutic strategies. Bone marrow-derived mesenchymal stem cells (hBMSCs) are able to differentiate into osteoblasts, and NORAD aggrandizes the proliferation and differentiation of hBMSCs, depicting that NORAD may be associated with fracture healing [11]. However, the detailed mechanism of NORAD in fracture healing is not completely understood.

In this research, NORAD was inferred to be correlated with fracture healing. Patients with brittle fractures were selected to examine the expression of NORAD. The expression of NORAD was tested during the progression of fracture healing. Furthermore, the impacts of NORAD on proliferation, differentiation, and apoptosis of mouse osteoblast cell line (MC3T3-E1) were analyzed.

## 2. Materials and Methods

### 2.1. Patient Recruitment and Sample Isolation

A total of 87 patients with brittle fractures treated in BinZhou Medical University Hospital were recruited in this study, including 47 patients with hand fractures and 40 patients with intraarticular fractures. The patient's group included 42 males and 45 females with an average age of 65.19 ± 8.71 years old. In addition, 43 healthy participants were recruited as healthy controls. There were 21 males and 19 females in the control group with a mean age of 64.40 ± 9.18 years old. Exclusion criteria for patients were as follows: (1) younger than 18 years old, (2) malignant tumor, (3) inflammatory arthritis, (4) heart failure, kidney failure, and (5) autoimmune diseases. An approvement by the ethics committee of BinZhou Medical University Hospital was sought, and an informed consent form was signed by each participant. Blood samples of 5 ml were collected from each patient within 24 hours after fractures, 7 days, 14 days, 21 days, and 28 days after standardized fixed treatment. The blood sample was allowed to stand for more than half an hour and centrifuged at 3500-4000 rpm for 5-10 minutes to get the serum. Serum specimens were deposited at -80°C for later use.

### 2.2. Cell Incubation and Management

All MC3T3-E1 cells were purchased from Shanghai Cell Bank, Chinese Academy of Sciences, and cultured in the alpha-minimum essential medium (HyClone, USA) containing 1% penicillin-streptomycin (Sigma-Aldrich, USA) and 10% fetal bovine serum.

The oligonucleotide sequences of NORAD from GenePharma (Shanghai, China) were cloned into pcDNA 3.1 vectors to build overexpression carriers. Besides, the si-NORAD from Gene Pharma was used to interfere with normal NORAD expression. According to the manufacturer's instructions, instantaneous transfection of synthetic molecules was carried out using Lipofectamine 3000 reagent (Invitrogen, USA). All following experiments were conducted after two-day incubation.

### 2.3. RNA Extraction and Detection

TRIzol LS reagent (Invitrogen, USA) was added to serum and cells, and total RNA was isolated and extracted. For the NORAD, the first-strand cDNA synthesis mixture of Hifair (Xiasheng, China) was used to synthesize the cDNA. For miR-26a, the total RNA was synthesized into cDNA by using an miRNA strand 1 cDNA synthesis kit (Lianmai Bio, China). Then, an miRNA qPCR kit (Lianmai Bio, China) was used to amplify the cDNA sample of miR-26a by qRT-PCR. The qRT-PCR was used to amplify cDNA samples of NORAD with qPCR premix (Lianmai Bio, China). The relative expression was calculated by the 2^-∆∆CT^ method. U6 and *β*-actin were used as internal reference genes.

### 2.4. Detection of MC3T3-E1 Cells' Proliferation, Differentiation, and Apoptosis

At 0, 24, 48, and 72 hours after cell treatment, the proliferation of MC3T3-E1 was evaluated by MTT (Saint-Bio, Shanghai, China). About 5 × 10^4^ cells were spread in 96-well plates, then 20 *μ*l MTT reagent was added and incubated at 37°C for 4 hours. Following that, 150 *μ*l Formanzan reagent was added. After being incubated for 4 hours, the absorbance of each well was measured at 570 nm.

Cells were cultured in a humid environment containing 5% CO_2_ at 37°C. Bone morphogenetic protein 2 (BMP2) was used for the differentiation induction of MC3T3-E1 cells. MC3T3-E1 cells were inoculated into a 6-well plate with a density of 10^6^ cells per well and cultured in the medium containing 200 ng/ml BMP2 for 14 days, and the medium was refreshed every 2 days. The differentiation of MC3T3-E1 cells was reflected by the levels of alkaline phosphatase (ALP), runt-related transcription factor 2 (Runx2), collagen 1, and osteopontin (OPN). ELISA kits from Elabscience Biotechnology (Wuhan, China) were utilized for the identification of cellular differentiation after cells being differentiated for 14 days.

Cells were incubated for 24 hours and digested with trypsin free of EDTA. The cells were collected and washed twice with phosphate-buffered saline (PBS). After centrifugation for 5 min, the supernatant was discarded, and 195 *μ*l Annexin V-FITC binding solution was added to resuspend the cells. A total of 5 *μ*l annexin V-FITC and 10 *μ*l propidium iodide (PI) were added to each well, and the plates were incubated in the dark for 10-20 minutes at room temperature. The fluorescence intensity was detected by flow cytometry. The kit used in this experiment was the Annexin V-FITC apoptosis detection kit (Beyotime, China).

### 2.5. Luciferase Activity Assay

The target relationship between miR-26a and NORAD was detected by a double luciferase reporter gene detection kit (Yeason, China). Before detecting the relationship between miR-26a and NORAD, the pmirGLO vector was transfected with wild-type (WT) or mutant (MUT) 3′-UTR of NORAD to build WT-NORAD or MUT-NORAD vectors. After cloning, the two plasmids were transfected into cells together with miR-mimic, miR-inhibitor, mimic-NC, or inhibitor-NC, respectively. After transfection, these cells were lysed. Then, 100 *μ*l of the sample was mixed with 100 *μ*l of luciferase detection reagent, and the relative luciferase activity was measured by a chemiluminescence instrument.

### 2.6. Statistical Analysis

GraphPad 9 was used to analyze the data. Student's *t*-test and one-way ANOVA were used for comparison between groups. *P* < 0.05 is used to demonstrate the statistically significant difference.

## 3. Results

### 3.1. Abnormal Expression of NORAD in Patients

The expression level of serum NORAD in patients with hand fracture and the intra-articular fracture was detected by qRT-PCR. The expression of NORAD in patients with hand fracture and the intra-articular fracture was both decreased compared with control individuals (Figure 1(a), *P* < 0.001). The expression of NORAD in male patients group and female patients group exhibited a similar tendency to that in total patients (Figure 1(b), *P* < 0.001). However, there was no difference in NORAD expression between female and male patients in control group, hand fracture group, and intra-articular fracture group (Figure 1(b), *P* > 0.05).

As seen from Figure 1(c), compared with the 1st day, the expression level of serum NORAD in patients with hand fracture healing increased gradually with time. Compared with the 1st day, there was no significant difference in serum NORAD expression in patients with hand fractures on the 7th day. On the 14th, 21st, and 28th days, the expression level of serum NORAD in patients with hand fractures increased significantly (*P* < 0.01). The same result was certified in the healing phase of patients with intra-articular fractures. On the 14th, 21st, and 28th days, the expression level of serum NORAD in patients with intra-articular fracture was significantly higher than those on the 1st day (Figure 1(d), *P* < 0.05). The results indicated that the imbalance of NORAD expression might change with the stage of fracture healing.

### 3.2. Roles of NORAD for MC3T3-E1 Cells

In addition, to investigate the effect of NORAD on fracture healing, NORAD was overexpressed or interfered with artificially. The level of NORAD was increased in the pCDNA3.1-NORAD group, and inhibited in the si-NORAD group, confirming that NORAD could be regulated by pCDNA3.1-NORAD and si-NORAD in vitro (Figure 2(a), *P* < 0.001).

An increase in MC3T3-E1's proliferation was found in the NORAD overexpression group, while interference of NORAD inhibited the cell proliferation (Figure 2(b), *P* < 0.001). Differentiation of osteoblasts is one of the important progression of bone formation, thus, we further confirmed whether NORAD was involved in osteogenic differentiation. We upregulated or downregulated NORAD in differentiated MC3T3-E1 cells and then detected the levels of osteogenic differentiation markers, including ALP, Runx2, Collagen I, and OPN. As shown in Figure 2(c), a high expression level of NORAD enhanced the levels of ALP, Runx2, Collagen I, and OPN, while a low expression level of NORAD suppressed the levels of ALP, Runx2, Collagen I, and OPN (*P* < 0.01). In addition, overexpression of NORAD prevented cell apoptosis, while reducing the expression level of NORAD led to the augment of cell apoptosis (Figure 2(d), *P* < 0.001).

### 3.3. Relationship of miR-26a with NORAD

To understand the detailed mechanism of NORAD in regulating fracture healing, we examined the target of NORAD in brittle fractures. Bioinformatics program exhibited that miR-26a had binding sites with the 3′UTR of NORAD (Figure 3(a)).

After cotransfection of the miR-26a mimics or miR-26a inhibitors with NORAD-WT 3′UTR, luciferase activity was significantly inhibited or increased (Figure 3(c), *P* < 0.001), while the luciferase activity in NORAD-MUT group was unchanged (Figure 3(b), *P* > 0.05). Increasing NORAD suppressed miR-26a levels, whereas inhibiting NORAD exerted the opposite function (Figure 3(c), *P* < 0.001).

### 3.4. Expression of miR-26a in Patients with Fracture

The ascended expression of miR-26a was identified in patients with hand fracture and intra-articular fracture (Figure 4(a), *P* < 0.001). In different gender groups, the expression of miR-26a was elevated in patients with intra-articular fracture and hand fracture (Figure 4(b), *P* < 0.001), while no discrepancy was found on miR-26a levels due to the gender difference (Figure 4(b), *P* < 0.05). Additionally, the opposite tendency of NORAD expression and miR-26a expression was found in inpatients with hand fracture (Figure 4(c), *P* = −0.752, *P* < 0.001) and intra-articular fracture (Figure 4(d), *P* = −0.764, *P* < 0.001). In both hand fracture and intra-articular fracture, the expression of miR-26a was lessened with the fracture healing (Figures 4(e) and 4(f), *P* < 0.05). All the above results further confirmed that miR-26a directly targets NORAD in fracture.

## 4. Discussion

Fractures are common traumatic damages, and nonunion and delayed union of fractures impose a severe economic and mental burden on patients [12]. The incidence of brittle fractures increases every year, probably due to a sedentary lifestyle, vitamin D deficiency, and an increased fall in the elderly population [13, 14]. Osteogenic proliferation and bone regeneration are chronic and intricate biological procedures, which are mediated by inherited and epigenetic indicators [15]. But the elements in osteogenic differentiation and osteogenesis are unsettled.

Accumulating evidence prove that lncRNAs may broadly contribute to tuning the expression pattern of specific downstream genes [16]. Several progressions, like osteogenesis, fracture repair, and bone remodeling are controlled by lncRNAs [17–19]. Behera and colleagues report that lncRNA H19 participates in microstructural changes of bone in an immunocompromised nude mouse model [20]. lncRNA MALAT1 accelerates osteoblast activity via miR-34c in mesenchymal stem cells, suggesting lncRNA as promising novel modulators amid bone formation [21]. Much attention is paid to the impacts of NORAD on several disorders. High NORAD expression in colorectal cancer is related to the advanced tumor stage [22]. In acute myocardial infarction, NORAD knockdown inhibits infarct size and fibrosis in a rat model [23]. In this recent study, the expression of NORAD was inhibited in patients with fractures and increased with the progression of fracture healing. These findings of qRT-PCR indicated that NORAD was involved in the fracture situation. The proliferation, differentiation, and apoptosis of osteoblast are essential parts influencing fracture repair and healing [24]. The overexpression of NORAD was attributable to the promotion of cell proliferation and differentiation and declined cell apoptosis, indicating that NORAD is a beneficial molecular in osteoblast activity. A previous investigation pinpoints that NORAD is lessened in osteonecrosis of the femoral head [11]. In short, the above findings established a connection between NORAD and fracture healing.

Most lncRNAs are pertinent to the regulation of miRNAs, and lncRNAs can reduce miRNAs' regulatory effect on mRNAs by acting as miRNA sponges [25]. lncRNA HAGLR/miRNA-19a-3p regulatory axis promotes the recovery of femoral neck fracture [26]. lncRNA HOXA11-AS serves as a sponge of miR-124-3p in fracture recovery [27]. In this research, miR-26a was found as a ceRNA of NORAD, and the luciferase activity report identified this finding. In addition, the overexpression of NORAD reduced the concentration of miR-26a, and the elimination of NORAD accelerated the quantity of miR-26a. In psoriasis and head and neck squamous cell carcinoma, NORAD negatively manages miR-26a [28, 29]. NORAD mediates hypertrophic scar formation by inhibiting the expression of miR-26a [30]. Moreover, knowledge of the correlations of miRNAs during fracture healing is widely presented by researchers [31]. The relative quantification of miR-26a was tested in patients suffering fractures. The findings pinpointed that miR-26a was highly expressed in patients with hand fracture and intra-articular fracture, suggesting the involvement between miR-26a and fracture. The negative correlations between miR-26a and NORAD were certified in patients with hand fracture and intra-articular fracture, further implying the interplay between miR-26a and NORAD. Further research on animal model of fracture is necessary for analysis of mechanism related to fracture healing.

## 5. Conclusions

Taken together, the expression of NORAD was diminished in patients with fractures and gradually fractured during the fracture healing. Enforced NORAD expression exerted a beneficial function on fracture recovery by promoting osteoblastic proliferation and differentiation and inhibiting apoptosis of MC3T3-E1 cells. MiR-26a is a ceRNA of NORAD in fracture. Fracture was conducive to the increment of miR-26a. A reverse trend of miR-26a expression and NORAD expression was pinpointed in this research.

## Figures and Tables

**Figure 1:** The expression of NORAD in patients with brittle fractures. (a) The decreased NORAD in patients with hand fracture and intra-articular fracture. (b) The expression of NORAD in male and female patients with brittle fractures. (c) Increased NORAD in patients with the fracture healing of hand fracture. (d) The expression of NORAD was gradually increased during the fracture healing in patients with intra-articular fracture. ∗*P* < 0.05, ∗∗*P* < 0.01, ∗∗∗*P* < 0.001.

**Figure 2:** Functions of NORAD in osteoblasts. (a) The regulation of NORAD expression with different transfections. (b) The proliferation of osteoblasts was regulated by NORAD. (c) Highly expressed NORAD increased osteoblastic differentiation, and lowly expressed NORAD inhibited increased osteoblastic differentiation. (d) Elevated apoptotic cells were found in the si-NORAD group and inhibited apoptotic cells in the pCDNA3.1-NORAD group. ∗*P* < 0.05, ∗∗∗*P* < 0.001.

**Figure 3:** miR-26a was a ceRNA of NORAD. (a) The putative binding bases between NORAD and miR-26a. (b) The findings of the luciferase report assay identified the targeted relationship between NORAD and miR-26a. (c) The expression of miR-26a was changed with the levels of NORAD. ∗∗∗*P* < 0.001.

**Figure 4:** The alternation of miR-26a expression in fracture. (a) The elevated expression of miR-26a in patients with brittle fractures. (b) The expression of miR-26a in different gender group. (c) NORAD levels were linked to the expression of miR-26a in patients with hand fractures. (d) NORAD was attributable to the reduced miR-26a expression in patients with intra-articular fractures. (e, f) The alternation of miR-26a with the fracture healing. ∗∗∗*P* < 0.001.

## Data Availability

The data used to support the findings of this study are available from the corresponding author upon request.
